The article "Listerial Meningitis and Brain Abscess With Coexisting COVID-19 Infection in a Young, Immunocompetent Male: A Case Report" was retracted in 2023. Reason: plagiarism.

# Listerial Meningitis and Brain Abscess With Coexisting COVID-19 Infection in a Young, Immunocompetent Male: A Case Report

**DOI:** 10.7759/cureus.29455

**Published:** 2022-09-22

**Authors:** Syed Faqeer Hussain Bokhari, Huma Sattar, Shaun Abid, Syeda Rabab Jaffer, Samar Sajid

**Affiliations:** 1 Medicine and Surgery, Mayo Hospital, Lahore, PAK; 2 Internal Medicine, Sharif Medical & Dental College, Lahore, PAK; 3 Internal Medicine, Allama Iqbal Medical College, Lahore, PAK; 4 Internal Medicine, Dow University of Health Sciences, Karachi, PAK; 5 Medicine, Dow University of Health Sciences, Karachi, PAK

**Keywords:** infectious disease, opportunistic infection, encephalitis, meningitis, brain abscess, listeriosis

## Abstract

*Listeria monocytogenes* (LM) is a gram-positive intracellular pathogen that can cause central nervous system infections such as meningitis, meningoencephalitis, rhombencephalitis, or cerebritis. It rarely causes a brain abscess. Listerial meningitis and brain abscess most commonly occur in immunocompromised individuals, neonates, pregnant females, alcoholics, and the elderly. We present a unique case of a young immunocompetent male who presented with listerial meningitis and brain abscess. Coexisting coronavirus disease 2019 (COVID-19) infection was also present. Since LM was not included in the differentials, the standard antibiotic regimen started for the meningitis therapy was ineffective. Remdesivir was administered to treat the coexisting COVID-19 infection. When the lumbar tap polymerase chain reaction pointed out that the causative agent was *Listeria*, we shifted to ampicillin and gentamicin therapy, to which the patient responded very effectively.LM is an atypical cause of meningitis and brain abscesses. A high index of suspicion is therefore required for early detection and effective treatment of listerial meningitis and brain abscess.

## Introduction

*Listeria monocytogenes *(LM) is an anaerobic, intracellular, gram-positive pathogen causing a dangerous foodborne disease, listeriosis [1]. LM is transmitted to humans via contaminated food products, especially soft cheese and deli meat. Immunocompromised individuals, alcoholics, pregnant women, neonates, and the elderly are more commonly infected [2]. Meningitis is the most common manifestation when the central nervous system (CNS) is involved [3]. Clinical signs of listerial meningitis are comparable to those of meningoencephalitis from other sources. Also, third-generation cephalosporins are ineffective as first-line therapy [4]. Only 1-10% of all listerial CNS infections and only 1% of all listerial infections lead to brain abscess [5]. This is an extremely rare scenario and its clinical manifestations lack specificity. Therefore, it is essential to be aware of this infection to start the treatment appropriately and get the best results [6]. 

We present the case of a 27-year-old immunocompetent male and despite the diagnosis of listerial brain abscess, no significant risk factors could be identified. This is a very unique case as it not only presented with one of the rarest CNS manifestations of listeriosis but also in a young, immunocompetent male. Only 20% of listerial brain abscess cases documented include individuals who have no known underlying risk factors [7]. We managed to successfully treat this case without surgical intervention via an antibiotic regimen of ampicillin and gentamicin. We also implore that in developing countries and settings where a lumbar tap is not possible, ampicillin should be co-administered with ceftriaxone and vancomycin in a case of meningitis, especially those that involve listerial risk factors. In such scenarios, inadequate treatment with cephalosporins or a late diagnosis of listerial infection can prove to be highly fatal.

## Case presentation

A 27-year-old male with a past medical history of migraine presented to the emergency department with severe headache, diarrhea, and semantic issues. He had been taking domperidone and paracetamol for two years on the recommendation of a friend as it helped him with migraine. The headache and diarrhea began four days prior to presentation; however, the patient had an acute change in mental status almost five hours before the emergency room visit, and as per the patient’s attendants, became more lethargic and less responsive. The patient was strictly vegetarian and did not consume any dairy products, eggs, or deli meat, especially in the last week. 

On admission, his temperature was 39.9^o^C, heart rate was 107 bpm, blood pressure was 147/92 mmHg, respiratory rate was 17 breaths/min, and oxygen saturation was 92% on room air. On physical examination, the patient was unresponsive to verbal stimuli but responsive to sternal rub and painful stimuli. A score of 12 was recorded according to the Glasgow coma scale (GCS). Kernig’s and Brudzinski’s signs were negative. Laboratory testing on admission was notable for a leukocyte count of 16.65 x 109/L (79.8% neutrophils, 10.4% lymphocytes, and 8.9% monocytes), sodium of 132 mg/dl, potassium of 3.0 mEql/l, a urinalysis with ketones and glucose and a positive severe acute respiratory syndrome coronavirus 2 (SAR-COV-2) polymerase chain reaction (PCR) from nasal swab. The results of the human immunodeficiency virus (HIV) screening test was negative.

Computed tomography (CT) scan of head without contrast revealed heterogeneous attenuation in the left basal ganglia and inferior frontal lobe with surrounding vasogenic edema and a 3 mm midline shift. A brain abscess was suspected. In the emergency department, the patient was given acyclovir 1000 mg intravenous piggyback (IVPB), cefepime 2g IVPB, vancomycin 1g IVPB, ketorolac 15mg IVPB, and 1 liter of lactated ringers. After discussion with neurology, the decision was made to defer a lumbar puncture at the time given the CT findings of midline shift with questionable mass. Given the patient’s septic presentation, encephalopathy along with the CT findings concerning meningitis/encephalitis, the patient was admitted for further evaluation and management. Following the therapy, the patient’s mental status mildly improved and he was aware of time, space, and person; however, he was still intermittently lethargic. The sodium levels of the patient decreased from 132 mEq/l to 124 mEq/l, and he was started on hypertonic 3% saline. The neurologist assessed the patient and noted the patient had diminished strength of the right upper extremity with a right facial droop and recommended performing an MRI of the head with and without contrast to evaluate for brain abscess as well as consulting a neurosurgeon regarding the possible brain abscess. The neurosurgeon recommended continuing the antibiotics, and follow-up cultures; however, no neurosurgery intervention was recommended at the time. The infectious disease specialist recommended continuing empiric antibiotics ceftriaxone and metronidazole and to follow up with an MRI head with contrast. The MRI head showed a heterogeneous lesion centered within the left basal ganglia and thalamus with mass effect on the left lateral ventricle with mild left-to-right midline shift (Figure 1A). Blood culture from two sets of aerobic and anaerobic bottles grew LM. A lumbar puncture was performed on day two (Table 1) and the lumbar puncture PCR came back positive for LM*.* The antibiotics were then adjusted to ampicillin and gentamicin by the end of day two.

**Figure 1:** (A) FLAIR MRI brain at time of admission showing heterogeneous lesion centered within the left basal ganglia and thalamus with mass effect on the left lateral ventricle with mild left-to-right midline shift; (B) FLAIR MRI brain taken 1.5 months later showing significant improvement in edema with decreased mass effect and resolution of midline shift. FLAIR: fluid-attenuated inversion recovery

**Table 1:** Results of preliminary investigation of CSF. CSF: cerebrospinal fluid; PCR: polymerase chain reaction

Investigations	Results	Normal Values
CSF Appearance	Clear	Clear
CSF Color	No color	No color
Total Nucleated Cell Count, CSF	80	0-5 (u/L)
CSF Segmented Neutrophils	22	0-6%
CSF Lymphocytes	14	40-80%
CSF Monocytes/Macrophages	44	15-45%
Protein, CSF	72	15-45 mg/dl
Glucose, CSF	73	40-70 mg/dl
Culture, CSF	No growth	No growth
Gram Stain, CSF	No organisms seen, no WBCs seen	No organisms seen, no WBCs seen
CSF PCR	*Listeria monocytogenes* detected	Not detected

Following the antibiotic adjustment, the patient’s mental status continued to improve and he was alert to self, place, and time and able to move extremities. There was mild stiffness of extremities and a persistent right facial droop. The patient’s hyponatremia improved. Levetiracetam 500mg twice a day was started as per neurology recommendation given MRI findings. Electroencephalography (EEG) showed mild left hemisphere slowing and occasional sharp frequencies over left posterior regions suspicious of underlying hyperexcitability. The infectious disease recommendation was to continue ampicillin 2 g IV every four hours and gentamicin 140 mg IV every eight hours.

The patient continued to do well and was discharged home on day six to continue his IV course of antibiotics ampicillin and gentamicin. A repeat MRI brain was performed approximately five weeks after discharge and showed significant improvement in edema and signal abnormality involving the left corona radiata, external capsule, and left basal ganglia/thalamus with decreased mass effect and resolution of midline shift (Figure 1B). 

## Discussion

LM can infect tissues that are otherwise relatively immune to infection such as gravid uterus, fetus, and CNS. It can infect both the meninges and parenchyma of the brain. CNS manifestations include meningoencephalitis, rhombencephalitis, and cerebritis [3]. In rare cases, it may lead to brain abscess [8]. Compared to other types of brain abscesses, listerial brain abscesses usually affect the brainstem unilaterally involving medulla oblongata and pons followed by supratentorial white matter and cerebellar hemispheres [9,10]. In our case, subcortical grey tissue including the thalamus and basal ganglia was involved. According to Zhang et al., statistical evaluation of 84 cases from 1968 to 2020, the mean age of patients who developed listerial brain abscess was 52.9 and 61.9% of these were males. The mortality rate was 25% and the probability of obtaining positive blood or CSF culture was 69.1% [6]. In our case, blood culture and lumbar tap PCR were positive; CSF culture was negative.

The bacteria may enter CNS via hematogenous spread from the digestive tract [11]. The choroid plexus epithelium gives LM access to the CNS and results in a meningitis infection [12]. On the other hand, the cerebral capillary endothelium may allow LMto enter the brain parenchyma. It may travel retrogradely through the neurons to the brain and enter CNS. The pathogenic cause of the classic multi-tubular look of listerial brain abscess on imaging, also known as “tunnel-sign” or “worm-like appearance” is attributed to the axonal invasion of LM [13]. It has also been suggested that LM-infected macrophages may enter the middle cerebral artery via endothelial cells, causing cerebritis, which results in the development of brain abscesses [14]. Since the defense mechanisms against LM involve cell-mediated immunity hence immunocompromised individuals such as HIV-infected patients are more prone to listerial brain abscess. However, in our scenario, the patient was immunocompetent and in a perfect state of health prior to infection.

LM has a non-specific clinical appearance that is comparable to bacterial or viral meningitis. Symptoms include fever, headache, vomiting, diarrhea, and altered mental state [15,16]. Brain abscess is usually visualized on MRI of head. Depending on the patient’s age and comorbidities, several empiric therapies for bacterial meningitis are suggested. *Streptococcus pneumoniae*, *Neisseria meningitidis*, and LM are the most frequent etiologies [17].* Neisseria meningitidis* and *Streptococcus pneumoniae* are the most probable pathogens to infect children and people aged 2 to 50 years, and vancomycin and ceftriaxone would be the first line of treatment. LM is not usually included in the list of potential pathogens until the patient population is over 50, has impaired cellular immunity, or has alcoholism; only then ampicillin is included as an empiric treatment together with vancomycin plus ceftriaxone [18].

## Conclusions

Given the rarity of brain abscesses and the lack of clear guidelines for the best course of treatment, the kind and length of therapy, we think it is imperative to conduct further research on this complication. Immunocompetent patients should also be suspected of having LM infection, and novel molecular biology tools are crucial in the early detection of this uncommon condition. Since our patient was young and immunocompetent, ampicillin was not strictly necessary to provide *Listeria *coverage. However, we advise that ampicillin should be added to the regimen in case of meningitis with coexisting brain abscess, especially in developing countries and settings where a lumbar tap is not feasible.
